The article "Efficient Liver Segmentation from Computed Tomography Images Using Deep Learning" was retracted in 2023. Reasons: signs of a paper mill; compromised peer review; unreliable results or conclusions.

# Efficient Liver Segmentation from Computed Tomography Images Using Deep Learning

**DOI:** 10.1155/2022/2665283

**Published:** 2022-05-18

**Authors:** Mubashir Ahmad, Syed Furqan Qadri, M. Usman Ashraf, Khalid Subhi, Salabat Khan, Syeda Shamaila Zareen, Salman Qadri

**Affiliations:** ^1^College of Computer Science and Software Engineering, Computer Vision Institute, Shenzhen University, Shenzhen, Guangdong Province 518060, China; ^2^Department of Computer Science and IT, The University of Lahore, Sargodha Campus, 40100, Lahore, Pakistan; ^3^Department of Computer Science, GC Women University, Sialkot 51310, Pakistan; ^4^Department of Computer Science, King Abdulaziz University, Jeddah 21589, Saudi Arabia; ^5^Faculty of Information Technology, Beijing University of Technology, Beijing 100124, China; ^6^Department of Computer Science, MNS University of Agriculture, Multan 60650, Pakistan

## Abstract

Segmentation of a liver in computed tomography (CT) images is an important step toward quantitative biomarkers for a computer-aided decision support system and precise medical diagnosis. To overcome the difficulties that come across the liver segmentation that are affected by fuzzy boundaries, stacked autoencoder (SAE) is applied to learn the most discriminative features of the liver among other tissues in abdominal images. In this paper, we propose a patch-based deep learning method for the segmentation of a liver from CT images using SAE. Unlike the traditional machine learning methods, instead of anticipating pixel by pixel learning, our algorithm utilizes the patches to learn the representations and identify the liver area. We preprocessed the whole dataset to get the enhanced images and converted each image into many overlapping patches. These patches are given as input to SAE for unsupervised feature learning. Finally, the learned features with labels of the images are fine tuned, and the classification is performed to develop the probability map in a supervised way. Experimental results demonstrate that our proposed algorithm shows satisfactory results on test images. Our method achieved a 96.47% dice similarity coefficient (DSC), which is better than other methods in the same domain.

## 1. Introduction

Segmentation of a liver is an essential step in different types of medical uses such as liver diagnoses, transplantation, and tumor segmentation [1, 2]. Due to the huge variation in the liver contour, the same intensity level in neighboring organs, low contrast, linkage of tissues, and various organs is overlapped which are the leading challenges in liver segmentation. In the previous few decades, a combination of techniques has been suggested for the segmentation of a liver from CT images. The details of different methods are given with pros and cons in the literature [3, 4]. Various techniques have been suggested for the segmentation of a liver which are graph cut [5, 6], level set [7, 8], thresholding [9], and region growing [10]. Preventing under-segmentation and boundary leaks are the big issues in gray-level techniques where the intensity in different organs.

Normally, initialization of automatic methods with morphological operations and certain thresholds to handle these problems [11] while semiautomatic approaches with minor user initialization and interaction can get the best results. J. Peng et al. [12] proposed a semiautomatic technique that used blood vessels for the segmentation of a liver using CT images. Another method [13] is the mixture of combined intensity, surface smoothness, and regional appearance to handle the fuzzy boundaries and in-homogeneous background [14], while these methods have promising outcomes but the selection and user initialization are the primary disadvantages. Model-based techniques are robust where the representative liver contour is utilized to deal with the problem of segmentation. Some existing model-based methods have been reported previously which rely on the statistical shape model (SSM) [15–17]. Large dissimilarities in the liver contour with a small dataset are a real task for SSM-based techniques. To overcome this problem, sometimes, a combination of SSM is utilized with deformable models [18, 19] or integrated with the level set method [20] to overcome the problem. Dictionary learning [21] and sparse shape composition (SSC) [22, 23] were used to plan an improved method that deals with the liver shape having complex variations. Atlas-based methods [24] registered the multiatlases or a single Atlas having a reference image and deformed the Atlas image by combining the labels. Therefore, these techniques are not very simple because of the huge variation in the shape of a liver that depends on the process of registration. In addition, the complications in Atlas computation and selection are proposed in the recent methods [25, 26]. Measurement of the blood vessel is performed with the thresholding segmentation method [27]. All the above techniques are semiautomatic and need user interaction in some way which is a drawback of these methods.

In recent years, progressive research based on automatic methods done in the field of computer vision and image processing using deep learning. Deep learning has three main building blocks which are stacked autoencoder (SAE), deep belief network (DBN), and convolutional neural network (CNN). CNN has been used in multiple tasks such as the classification of images [28] and recognition of visual objects [29]. For the segmentation of knee cartage, it is applied and found a very useful application in the medical image processing field [30–32]. CNN revolutionized natural imaging by learning high-level features [33–35], but it can only train labeled data in large amounts which is a drawback of this method. Recently, many researchers presented the results in medical image segmentation using deep learning methods [36–42]. Liver segmentation from SAE has been proposed [43], while DBN has been used for the liver and vertebrae segmentation that prospers respectable results [44–46]. Vertebrae segmentation using stacked sparse autoencoder (SSAE) was applied to CT images and got efficient results [47–49]. For the classification of breast cancer in histopathological images with DBN has been proposed which got improved results [50]. For liver segmentation using CNN, a recent method is used to get reasonable results [51].

In our work, we use patch-based SAE to segment the liver from the abdomen in CT images. This method uses unsupervised feature learning in the pretraining where many layers are added to make the deep network. The contribution is as follows:

- Unsupervised features in pretraining were taken from multiple layers of autoencoders; then, these features are fine tuned with the labels of a given input image in a supervised way.
- These images are distributed into several patches, and each patch is given as an input to the network.
- The complexity of the system is very less because the proposed method accepts patches as input instead of the whole image.
- Recently, CNN-based liver segmentation methods need larger hardware resources, but the proposed method can train the model with very few hardware resources.
- We successfully got the best results with a limited number of resources (data and hardware).

The remaining part of the paper is structured as follows. Sections 2 and 5 of the paper describe the background work, methodology, experiments, and results, respectively; Sections 6 and 7 are about the discussion and conclusion of the paper.

## 2. Background Work

The proposed method [52] is presented in a workshop on high interaction components, and the subject of the method was a 3-D region growing criteria of nonlinear coupling where new voxels are included in the region of seed. If the neighborhood weighted intensity difference and intensity of seed is less than a given threshold, then the region grower method is utilized iteratively inside the liver at different locations, where this algorithm works for the entire region of the liver being segmented. Missing parts and leaked regions are corrected manually using a “virtual knife.” A user-specified cutting plane “Virtual Knife” removes all the labels from one side. Postprocessing is applied to extend the segmentation.

A region growing technique [53] is inspired by a localized contouring method with modified k-mean integration. In the first step, a modified K-mean algorithm [54] is used to divide the slice into five pieces from the CT image that is liver, peripheral muscles, surrounding organs, ribs, and outside of the body. Selecting the seed point for a k-mean algorithm is an important task, while a localized contouring algorithm is used to get the best shape of the liver. The localized contouring works dynamically around the liver to follow the point under consideration rather than its whole statistics, and the localized region growing algorithm is more powerful than the contouring algorithm [55]. Novel volume interest and intensity-based reggrowthwing are then utilized to complete the process of a single slice initialization [56]. In medical imaging, atlas-based segmentation is a way of analyzing images through their structure labeling or a set of frameworks. The main purpose of this method is to involve the radiologist in the process to discover the disease. The workflow of this approach is to optimize the medical images for the identification of significant anatomy [57]. The purpose of an Atlas is to make a reference set for the segmentation of new images. These methods consider the problems of registration to handle the problems of segmentation [58].

For the extraction of a liver from the abdomen, the level set method is used where the preprocessing is applied before the segmentation [59]. The removal of noise is performed in preprocessing phase and enhanced the contrast of the image using the average, Gaussian, and contrast fitting filters while the ribs boundary algorithm [59] enhanced the boundaries and segmented the whole liver using the level set method. In the postprocessing phase, the watershed approach is used for more stable results and well-connected boundaries. The 3-D level set method is proposed [60] in which a medium level of user involvement is used for the liver segmentation. The user requires selecting the 2-D image contours, and these contours are resampled in many directions where the preferred direction is orthogonal. On the liver, boundary contour points are placed and using cubic splines for interpolation. The radial basis function [61] is used to generate the smooth surface when the user sets 6 to 8 points. This smooth surface passes through all contours and interpolates all the images. This surface helps to create a geodesic active contour which is the same as the true liver boundary.

The gray level methods are presented [62–65] in which the histogram of the whole volume through the preset gray level range for the identification of liver peak having two thresholds [62]. The purpose of these thresholds is to determine a liver binary volume which is processed heavily to delete the organ through morphological operators. Through the canny edge detector, this binary volume is used for the selection of binary mask [66] where the boundaries lie in the external part of the liver. The edges which were previously selected are input to the gradient vector flow algorithm; this helps in the creation of the initial segmentation of a liver and then modification through snakes. The extension of the algorithm to the segmentation of a liver volume is a slice by slice manner where the adjacent slice is constrained by the preceding slices. For this aim, a user selects the initial slice, and then the other work is automatically done by the system. The contour of the liver is used as a mask for the detection and elimination of errors. At last, the snake algorithm and gradient vector flow are applied again to produce more accurate results.

The anatomic knowledge is captured and described which is based on the position, size, and shape of each organ of the abdomen where the deformable models and statistical models are very famous. The early work of the statistical model has been done [67] successfully, and enhanced work has been implemented [68, 69]. The variational framework algorithm proposed by Tsai et al. [70] is embedded in the work [71] where free deformation is used for the statistical shape model segmentation step, and 50 training samples were used to build the statistical model that is inspired by the signed distance function where nonpara metrical shape distribution is used which is based on density estimation [72]. The analysis of the image intensity histogram is carried out using a Gaussian mixture model for the initialization of SSM. From this analysis, the intensity of the liver tissue is reduced through the image threshold. To minimize the energy of segmentation, a gradient descent algorithm is used to find the boundary where nonrigid registration is utilized to refine the segmentation.

## 3. Materials and Methods

The proposed system is distributed into two parts that are training and testing, which are shown in Figure 1. The training patches from CT images are sent to the corresponding autoencoder for feature learning, and test images are sent to the trained model to segment the liver from CT images.

### 3.1. Preprocessing of Data

The vital part of image segmentation is preprocessing in which processed images are produced from raw CT images that can discriminate the features of the liver from the other organs in the human body. We enhanced the contrast and normalized the images using zero mean and unit variance for each image. Then, we applied a Gaussian noise that is helpful to make the edges obvious [73].  Figure 2 shows the preprocessing stages, that change the appearance of the image, and this process is done for the whole dataset. The utilization of a Gaussian noise can strengthen the edges of the image where we selected the mean value 0 and variance value 0.02.

All images are cropped at a certain point that does not disturb the liver area, and each image is distributed into patches where these patches are given as input to the system for training. In such a way, the patch is considered an elementary portion of learning in our research. Positive patches are the region or patch which is reserved from the area of a liver, and we consider it as a foreground. Therefore, negative patches are the sections that are occupied from the background as shown in Figure 3. When preprocessing is done, we processed the images for the remaining experiment. The network training is done with a class balancing where we extracted 400,000 patches where half patches are related to the foreground and the other half are related to the background. Patch size was 27 × 27 for the experimentation.

### 3.2. Training the Stacked Autoencoder

For feature learning, we are using the stacked autoencoder which is a deep learning inspired method where feature learning is an unsupervised manner in pretraining. Autoencoders possess three layers which are input, hidden, and output layers. The training of an autoencoder has two parts that are encoder and decoder. In each hidden unit, there is no connection with other neurons in the same layer and is connected to all neurons in each neighboring layer. The feed-forward propagation method with the sigmoid function is used to calculate the weighted sum of SAE.

(1) $$\begin{array}{c} f\left(x\right)=\frac{1}{\left(1+\exp\left(-x\right)\right)},\\ a^{2}=f\left(z^{1}\right)=f\overset{m}{\underset{i=1}{\sum }}w^{1\;}x^{1}+b^{1}, \end{array}$$

where *x* is the input to the network, w^1^ is the weight matrix for the input layer, b^1^ is the bias for the first layer, a^2^ is the activation values of the first layer, and z^1^ is the weighted sum obtained from the input layer. The purpose of a single autoencoder is to learn the more discriminative demonstration of the inputs, which evaluate the cost function. The following formula is used for this purpose:

(2) $$\begin{array}{c} J\left(W,b\right)=\frac{1}{m}\overset{m}{\underset{i=1}{\sum }}\left[\frac{1}{2}h_{W,b}\left(x\right)-x^{2}\right]+\frac{a}{2}\overset{2}{\underset{i=1}{\sum }}\overset{sl}{\underset{i=1}{\sum }}\overset{sl+1}{\underset{j=1}{\sum }}{\left(W_{ji}^{l}\right)}^{2},\\ h_{w,b}\left(x\right)=\;a^{3}=f\left(z^{3}\right), \end{array}$$

where W represents the whole matrix and *b* is the bias matrix of the network, *m* is representing the training cases, and ‘*a*' is a weight decay parameter. The goal of an encoder is to discover a suitable parameter matrix that produces the minimum value of *J* (W, b). The input demonstration of *x* is *h*_w,b_(x). Moreover, the gradient descent algorithm is used to search for the best solution

(3) $$\begin{array}{c} W^{1}=W^{1}-\beta \frac{\partial J\left(W,b\right)}{\partial W^{1}},\\ b^{1}=b^{1}-\beta \frac{\partial J\left(W,b\right)}{\partial b^{1}}. \end{array}$$

Here, W^1^ is the connecting weight matrix and *ß* is the learning rate of the autoencoder. When training of the first layer is completed, the outputs of the first layer are given to the second layer of the autoencoder, and the training process is the same as in the first layer. This process finished the 2 layers training successfully. We implemented the softmax regression as a classifier due to numerous reasons: (i) the training time of the softmax regression model is much less than other classifiers like SVM, and (ii) it has better scalability if we request the model to predict the liver among other organs in our case. Moreover, the training time is not increased when we want to predict more than one class using the softmax regression model. The following is the hypotheses function:

(4) $$\begin{array}{c} h\Theta =\frac{1}{1+\text{exp}\left(-\Theta^{T}x\right)}. \end{array}$$

Θ is the parameter of the softmax regression model which controls the gradient of the cost function as follows:

(5) $$\begin{array}{c} J\left(\Theta \right)=\frac{-1}{m}\left[\overset{m}{\underset{j=1}{\sum }}y^{i}\text{log}h_{\Theta }\left(x^{i}\right)+\left(1-y^{i}\right)\text{log}\left(1-h_{\Theta }\left(x^{i}\right)\right)\right]+\frac{\lambda }{2}\overset{k}{\underset{i=1}{\sum }}\overset{n}{\underset{j=1}{\sum }}\Theta_{ij}^{2}, \end{array}$$

where *m* represents the total number of training cases and *λ* is the weight decay term. The network is fine tuned as a whole, and we used the features first and the second layer of autoencoder with the corresponding labels. After the completion of pretraining, fine tuning is performed with a backpropagation neural network. Fine tuning is the way to decrease and improve the error rate in autoencoders. The training process of the model is given in Figure 4.

### 3.3. Postprocessing

The initial segmentation is performed through SAE-based classification model where the initial probability map has a problem of misclassified boundaries. There are holes in the liver surface in some slices where morphological operation is performed to fill the holes. We find out the largest blob in the image and remove other small misclassified pixels that appeared around the liver. To smooth the liver boundaries using morphological closing operations which can find the weaker pixels on the liver boundaries, these weak pixels are removed to get a smooth liver.

## 4. Experimentation

### 4.1. Dataset Selection

MICCAI-Sliver'07 is an openly accessible dataset having 20 3D images with ground truths of a liver. The number of 2D slices in each image is varying from 64 to 512. On the organizers of the MICCAI-Sliver'07 website, this dataset is freely available (http://sliver07.org) which has a combination of pathologies that are cysts, tumors of different sizes, and metastases. Using different scanners, each image is contrast-enhanced having an axial dimension of 512 × 512. MATLAB 2018b is used to complete this experiment with Intel Core i7-8565U, 1.80 GHz CPU, 2 GB NVIDIA GeForce MX250 GPU, and 32 GB of RAM.

### 4.2. Parametric Selection

After preprocessing, our model is used for the experimentation which is given below: Initially, weights and biases were fixed to zero, and then we performed experiments with the random search for the range of hyperparameters. It shows in the literature that experiments with random search experimentation are more robust for hyperparameter optimization. Random search reacquired less time for computation and performed better network training. All hyperparameters are not important for experimentation, so random search is the method to identify the best hyperparameters [74]. During the pretraining stage, we set the learning rate at 0.001, and a momentum of 0.9 was given to the system. Scholastic gradient descent (SGD) algorithm was used in pretraining. The size of the training data patches was 400,000 where a balanced number of patches were used for each class (liver or background). Moreover, 70% of data were used for training and the remaining 30% for validation. The 27 × 27 patch was converted into vector form, so the input size of 729 is given to the model for training. The flattering input is given to the first layer of the autoencoder (AE1), whereas the second layer of the autoencoder (AE2) was trained on the output of the first autoencoder. The initialization of the feed-forward neural network with weights and biases was used in pretraining with 2 hidden layers of 200–100, and the final layer was the classification layer having 2 neurons which are the output of the given model (background or foreground). During the pretraining, the SGD algorithm was used. Labels are given for each patch in the fine tuning stage where we set the learning rate and momentum to 0.0001 and 0.9, respectively. Moreover, the sparsity proportion was set at 0.05, and weight decay was 0.000025 in this experiment with backpropagation. For the prevention of overfitting, weight decay is being utilized. For training, Sigmoid activation function with a mini batch size of 64 was used.  Table 1 shows the learning parameters of the proposed model which took 4 hours for pretraining and 36 hours for fine tuning.

A backpropagation neural network is used for the training, and the mean squared error (MSE) criterion is applied for error measurement. During the training process, our training error reached 0.01384, and the validation error was reached at 0.01486 with 3000 epochs. After this error, no more convergence was detected. On different parameters, Figure 5 shows the training and validation error. A learning rate of 0.0001 generated a good result with softmax output. Our experiments found that a very low learning rate yielded better results.  Figure 5(a) shows the finest validation and training results with a learning rate of 0.0001 and softmax output. Figures 5(b) and 5(c) show the bad validation results where we stop the training at 800 and 1000 iterations, respectively, with learning rates of 0.001 and 0.01 with the sigmoid output layer.

## 5. Results

Before we go to the details of the segmentation results, some common statistical methods are helpful in performance measurement. True Positive (TP) means all the pixels which are associated with the liver. True Negative (TN) means all the pixels which are associated with the background. False Negative (FN) are pixels related to the liver but not classified as liver, and False Positive (FP) are those pixels that are related to the background but do not classify accurately as background. Dice similarity coefficient (DSC) is to measure the overlapping of two masks where 0 means no overlapping and 1 means perfect dice score. The following equation describes the DSC:

(6) $$\begin{array}{c} DS\;C=\frac{2TP}{2TP+FP+FN}. \end{array}$$

Jaccard similarity coefficient (JSC) is the method to compare the original mask with the mask we created from the model:

(7) $$\begin{array}{c} JSC=\frac{TP}{TP+FP+FN}. \end{array}$$

Sensitivity is the measurement of accurately identified positive pixels (liver pixels). The mathematical equation is as follows:

(8) $$\begin{array}{c} \text{Sensitivity}=\frac{TP}{TP+FN}. \end{array}$$

Specificity is the measurement of accurately identified negative cases (background pixels). Mathematically, it is written as follows:

(9) $$\begin{array}{c} \text{Specificity}=\frac{TN}{TN+FP}. \end{array}$$

Accuracy is the measurement of differentiation between positive and negative cases; it is written mathematically as follows:

(10) $$\begin{array}{c} \text{Accuracy}=\frac{TP+TN}{TP+TN+FP+FN}. \end{array}$$

To calculate the precision, the following mathematical equation is used:

(11) $$\begin{array}{c} \text{Precision}=\frac{TP}{TP+FP}. \end{array}$$

The standard deviation (SD) is a positive square root of the variance which shows the value that how much deviated from the mean value. The following formula is used to calculate the standard deviation.

(12) $$\begin{array}{c} \frac{\sqrt{X-{\bar{x}}^{2}}}{n-1}. \end{array}$$

If we have a distribution in which *X* is the value, $\bar{x}$ is the mean value of all the samples and *n* is the total number of distributions.

### 5.1. Segmentation Results

We are presenting the results in the following section using the above statistical methods. The results are based on the MICCAI-Sliver'07 dataset.  Table 2 shows the results of our model on 5 images having 700 2D slices that were not used in the training set.  Table 2 shows the results from the MICCAI-Sliver'07 dataset that our model produces the mean results of 5 cases with 700 2D slices. The sensitivity, specificity, and accuracy of the model were recorded at 96.68%, 95.82%, and 96%, respectively. Precision, JSC, and DSC were observed at 95.97%, 92.91%, and 96.47%, respectively. The standard deviation on DSC was recorded at 1.03 which means our segmentation results of all the testing cases are much closer.  Figure 6 represents the segmentation results of the proposed model. To understand Figure 6, each row has a 2D CT image taken randomly from the test set. Each column represents the results which are as follows: (a) is the original CT image, (b) is the original label, (c) is the segmentation result of our model, (d) is the result after postprocessing where our method refined the liver, and (e) is the overlapping of the original label with our model, and green color shows the original label and red color shows the segmentation results generated by our model.

## 6. Discussion

The proposed model is simple and robust as compared to the other deep learning and machine learning methods. It segments the liver slice by slice where one slice takes 9 seconds for the segmentation of a liver from a CT scan image. We trained our model using patches where each patch represents the foreground and background which helps to reduce misclassification. Pixel-by-pixel classification is more complex and time consuming because an end-to-end learning needs in pixel-based image recognition [75]. So, there is no need to learn features manually in our patch-based deep learning method. We have selected the best patch size for training which is useful against overfitting in segmentation. The training was performed on a small dataset and got promising segmentation results.  Table 3 shows the relative outcomes of the proposed model with other techniques.

To compare our results with recent techniques, our model got promising segmentation results on liver segmentation. In [76, 77], both the methods are semiautomatic and the user needs to select the seed points. It is necessary to involve the users. Hence, the performance of our method over these methods is better. Our method got a DSC of 96.47%, whereas these methods got 94.03% and 93%. Another deep learning method CNN-LivSeg [32] scored a DSC of 95.41% on the same dataset. DBN-DNN [44] is based on a deep belief network, a deep learning method that scored 94.80% DSC, so our method is better than the proposed method. DBN-DNN is not working well on images with tumors, and it ignores the tumor area. Our proposed model performs well on all the images with tumors or nontumors.

## 7. Conclusion and Future Work

In this work, we proposed a model for the segmentation of a liver from CT scan images. Among other abdominal organs, the proposed algorithm learned robust representation of the liver. Moreover, utilizing the strategy of patches instead of pixel-by-pixel learning reduces the misclassification rate. We got a 96.47% DSC score, which is better than other related methods for liver segmentation. In the future, we will focus on a more discriminative deep learning architecture for the neural network to overcome the liver detection problems with other big datasets which are publically available.

Our system has some limitations where we only apply this model to liver segmentation from CT scan images. In the future, we will apply the same model with more optimized parametric selection on other organs such as kidney segmentation, brain tumor segmentation, and liver tumor segmentation problems.

## Figures and Tables

**Figure 1:** The workflow of the proposed liver segmentation model.

**Figure 2:** Ambiguous borders in the raw image (Left). Contrast enhancement (Middle). Gaussian noise addition (Right).

**Figure 3:** Extraction of positive and negative patches from CT images.

**Figure 4:** Detection of a liver from the proposed model.

**Figure 5:** On different parametric (a) selection, the training (b) and validation (c) results of the proposed model.

**Figure 6:** Segmentation results of the proposed model. The green color indicates the original labels and the red color shows the results generated by our model.

**Table 1:** Learning parameter of stacked autoencoders.

Parameter name	Value
Iterations in pretraining	80
Iterations in fine tuning	3000
Learning rate in pretraining and fine tuning	0.001, 0.0001
The activation function in each hidden layer	Sigmoid

**Table 2:** Results of the proposed model on the MICCAI-Sliver'07 dataset.

Case	Sensitivity (%)	Specificity (%)	Accuracy (%)	Precision (%)	JSC (%)	DSC (%)
#1	97.56	97.78	97.66	97.96	95.61	97.75
#2	96.77	96.48	96.63	96.74	93.71	96.75
#3	96.97	95.24	96.15	95.78	92.99	96.15
#4	96.59	93.54	95.24	94.95	91.86	96.76
#5	95.51	92.87	94.34	94.42	90.40	94.95
Mean	96.68	95.82	96.00	95.97	92.91	96.47
SD	0.75	2.02	1.27	1.42	1.96	1.03

**Table 3:** Comparative results of the proposed model with other methods.

Methods	DSC (%)
[76] Random walker	94.03
[77] Graph-based random walker	93.00
[32] CNN-LivSeg	95.41
[44] DBN-DNN	94.80
Our method	96.47

## Data Availability

The data underlying the results presented in the study are available within the manuscript.
